This article has been retracted.

# Alpha-synuclein overexpression in the olfactory bulb initiates prodromal symptoms and pathology of Parkinson’s disease

**DOI:** 10.1186/s40035-018-0128-6

**Published:** 2018-09-28

**Authors:** Haichen Niu, Lingyu Shen, Tongzhou Li, Chao Ren, Sheng Ding, Lei Wang, Zhonghai Zhang, Xiaoyu Liu, Qiang Zhang, Deqin Geng, Xiujuan Wu, Haiying Li

**Affiliations:** 1 Department of Genetics, Xuzhou Medical University, Xuzhou, 221004 China; 2 Department of Epidemiology and Health Statistics, Xuzhou Medical University, Xuzhou, 221004 China; 3 Department of Neurology, Affiliated Yantai Yuhuangding Hospital of Qingdao University, Yantai, 264000 China; 4 College of Medicine, Institute for Behavioral Medicine Research, The Ohio State University, Columbus, OH USA; 5 Department of Neurology, Affiliated Hospital of Xuzhou Medical University, Xuzhou, 221004 China; 6 Department of Pathology, Xuzhou Medical University, Xuzhou, 221004 China

**Keywords:** Alpha-synuclein, Prodromal animal model, Parkinson’s disease, Olfactory bulb, Autophagy

## Abstract

**Background:**

Parkinson’s disease (PD) is a neurodegenerative disease characterized by intraneuronal Lewy Body (LB) aggregates composed of misfolded alpha-synuclein (α-syn). The spread of misfolded α-syn follows a typical pattern: starting in the olfactory bulb (OB) and the gut, this pathology is followed by the progressive invasion of misfolded α-syn to the posterior part of the brain. It is unknown whether the administration of human mutant alpha-synuclein (hm-α-syn, a human mutation which occurs in familial PD) into the OB of rats would trigger similar α-syn propagation and subsequently cause pathological changes in broader brain fields associated to PD and establish an animal model of prodromal PD.

**Methods:**

hm-α-syn was overexpressed in the OB of rats with an AAV injection. Then motor and non-motor symptoms of the SD rats were tested in different behavioral tasks following the AAV injection. In follow-up studies, pathological mechanisms of α-syn spread were explored at the histological, biochemical and micro-structure levels.

**Results:**

The experimental results indicated that hm-α-syn was overexpressed in the OB 3 weeks after the AAV injection. 1) overexpression of the Hm-α-syn in the OB by the AAV injection could transfer to wider adjacent fields beyond the monosynaptic scope. 2) The number of tyrosine hydroxylase positive cells body and fibers was decreased in the substantia nigra (SN) 12 weeks after AAV injection. This was consistent with decreased levels of the DA neurotransmitter. Importantly, behavioral dysfunctions were found that included olfactory impairment after 3 weeks, motor ability impairment and decreased muscular coordination on a rotarod 6 weeks after the AAV injection.3) The morphological level studies found that the Golgi staining revealed the number of neuronal branches and synapses in the OB, prefrontal cortex (PFC), hippocampus (Hip) and striatum caudate putamen (CPU) were decreased. 4) phosphorylated α-syn, at Ser-129 (pSer129), was found to be increased in hm-α-syn injected animals in comparison to controls that overexpressed GFP alone, which was also found in the most of LB stained by the thioflavine S (ThS) in the SN field. 5) A marker of autophagy (LC3B) was increased in serval fields, which was colacolizated with a marker of apoptosis in the SN field.

**Conclusions:**

These results demonstrate that expression of exogenous mutant α-syn in the OB induces pathological changes in the sensitive brain fields by transferring pathogenic α-syn to adjacent fields. This method may be useful for establishing an animal model of prodromal PD.

## Background

Parkinson’s disease (PD), a movement disorder characterized by bradykinesia, rigidity, rest tremor, and postural instability, is caused by the loss of dopaminergic neurons in the substantia nigra (SN) and the appearance of intracellular inclusions, named Lewy bodies (LB), in the remaining neurons [1, 2]. There is a loss of 60–80% of the striatal or putaminal dopaminergic neurons before PD motor symptoms emerge [3, 4]. Currently, it is impossible to cure this disease.

Significant dysfunctions in the central nervous system in PD are thought to persist for several years before the onset of the classical motor syndrome, defining the prodromal phase. The prodromal phase in PD is a crucial period in the disease progression and is characterized by non-motor symptoms such as autonomic disturbances, depression, sleep disorders and, interestingly, olfactory dysfunction [5, 6].

Alpha-synuclein (α-syn) is a presynaptic nerve terminal protein, which represents 1% of the cytosolic protein in the brain [7]. Although the function of alpha-synuclein is not well understood, studies suggest that it plays a role in maintaining a supply of synaptic vesicles in presynaptic terminals by clustering synaptic vesicles, which help regulate the release of dopamine that is critical for controlling the start and stop of voluntary and involuntary movements [7].In the native form, it has a tertiary structure that resists aggregation, but the mutant α-syn exhibits no stable tetramer formation and is prone to aggregation [8]. Previous studies have indicated that α-syn was altered by various covalent post-translational modifications leading to changes in its folding and undergoes interneuronal transfer by limiting α-syn flexibility, modifying membrane association, limiting complex formation, and altering its degradation [9]. In PD, it is found that more than 90% of α-syn in the LB is phosphorylated on Ser-129, which has been commonly used as a marker of α-syn aggregation [10–12].

Recent studies have shown that α-syn mutations at A53T and A30P are related to a genetically transmitted or familial PD. This finding is the basis of a generation of transgenic animal models of PD [13, 14]. Also, recent publications suggested that α-syn can self-assemble to become a large aggregation, up to the size of an LB [15, 16]. Moreover, Braak et al. hypothesized that misfolded α-syn could be propagated from cell to cell similar to the pathological spreading of LB in sporadic PD, in which α-syn was converted into an abnormal aggregation [17–19]. This spreading pathology has been mimicked in experimental animals by injecting fibril α-syn and brain homogenates from transgenic mice or patients [20–22]. However, fibril α-syn is not a native protein of the brain and was produced in vitro after sonication [23]. Therefore, a model to recreate the physiological and pathological conditions seen in vivo is needed. Previous studies reported that mutant α-syn (A30P, A53T), as compared to wild-type α-syn, readily aggregates in vivo [24]. This suggests that the overexpression of a double point mutant (A30P, A53T) of human α-syn (hm-α-syn) might be used to mimic pathological conditions.

A stereotypical pattern of LB distribution has been found in PD, which appears to always start in the olfactory bulb as the first site of α-syn deposition in the CNS [17, 25, 26]. In parallel, olfactory deficits present as a leading prodromal symptom in clinical PD. Previous studies indicate that about 80% of PD patients have abnormal olfactory evoked responses, i.e., a decreased odor detection threshold, impaired odor identification, and reduced volume of the olfactory bulb [27–29]. However, it is unknown if the α-syn double mutant expression in the OB can trigger PD-like brain pathology beyond the monosynaptic level, particularly in regards to the dopaminergic system.

Glycoprotein (G)-deleted rabies virus (RV*dG*) has been a powerful and widely adopted tool for the study of the neural organization at the monosynaptic level. In these studies, RV*dG* and pseudotypes with EnvA were used to target rabies virus infections to a specific starter locus and were found to trans-synaptically label only direct presynaptic inputs throughout the mammalian brain [30]. With this approach, the Glycoprotein is deleted from the rabies genome and replaced by a transgene, such as GFP. As such, RV*dG* infections are restricted to where the Glycoprotein is provided and can only undergo retrograde spread across synapses to infect directly contacted presynaptic neurons [31]. This suggests that an *RVdG* based adeno-associated virus (AAV) vector can be packaged with the human double mutant α-syn (hm-α-syn) gene to express the hm-α-syn protein in a directed location with limited spread of the viral vector. As such, we hypothesized that expression of double mutant α-syn from a viral vector in the OB of rats would induce the sequential progression of Lewy Body-like pathology and induce selective dopamine loss beyond the monosynaptic scope of the vector.

In this study, we explored whether the expression of double mutant α-syn in the OB induced the following four aspects of PD: 1) pathology outside of the OB; 2) a close association between α-syn aggregation distribution and synaptic connectivity with the OB; 3) the aggregation of α-syn in regions without mutant α-syn expression; and 4) pathological changes in dopaminergic neurons. The results confirm that injections of AAV-hm-α-syn into the rat OB induced a novel model of prodromal PD that can be used to test new compounds designed to prevent or slow PD development.

## Methods

### Animals

Two-month-old male Sprague-Dawley rats (weight: 180-220 g, *n* = 50) were purchased from the Xuzhou Animal Centre and housed four rats per cage under 12 h light/dark cycle with free access to food and water. All experimental procedures were performed by the National Institutes of Health (NIH) Guide for the Care and Use of Laboratory Animals. All procedures performed were approved by the Animals Ethics Committee of Xuzhou Medical University. Efforts were made to minimize the number of animals used and their suffering. The number used in the experiment was approved by the Animals Ethics Committee of Xuzhou Medical University.

### AAV preparation and stereotaxic injection for overexpression of α-Syn

In the overexpression of α-Syn, AAV1/2 was used as a viral vector to deliver the cassette *CMV -syn -ires -GFP* that overexpresses the double-point mutation of human α-Syn (A30P and A53T: hm-α-syn) and GFP simultaneously. AAV 2/1 *-CMV -GFP* was used as a control. The human mutant cDNA of α-syn was gifted by Dr. Shujiang Shang (Peking University). The α-syn cDNA was inserted between the *CMV* promoter and the IRES element of pTR-UF12 to derive the construct. Vigen Biosciences company (Qingdao, China) finished AAV packaging and purification. An equivalent number of genome copies was determined using real-time quantitative PCR (4 × 1013 genome copies/μl) and collected.

Rats were anesthetized with ketamine (10 mg/ml) and 400 mg/kg chloral hydrate (4% in saline, 5 ml/kg, i.p.) and maintained with smaller doses (100 mg/kg) added every hour. All operations were performed on a heating pad. A small hole in the rats’ skulls was opened with a dental drill. The injection coordinates for the OB were 7.08 mm anterior to bregma, 1.0 mm medial-lateral, and 4.0 mm dorsal-ventral (Paxinos and Watson, 6th edition). The virus was placed at room temperature for 10 min before injection. Then the AAV was injected through a 27-gauge cannula connected to a 26-gauge I.D. polyethylene tubing and then to a 10-ul Hamilton syringe (Product Code: 4307205) mounted to a CMA/100 microinjection pump. The pump delivered 500 nl over 10 min to each side of the brain, and then the needle remained in place for an additional 10 min. The cannula was removed slowly (over 5 min) and the skin was sutured. After recovery from the surgery, rats were returned to their home cage.

### Detection of monosynaptic connectivity in the OB

To detect if theα-Syn overexpression in the OB is beyond the monosynaptic connectivity in the OB, the independent animals (*n* = 6) was used to detect monosynaptic connections in the OB by the rabies viruses (RV). For the RV, the titer of RV-EnvA-ΔG-dsRed was about 2 × 10^8^infecting unit per milliliter. For AAV viruses, the AAV9-EF1a-floxed-EGFP, AAV9-EF1a-Dio-GFP-TVA, and AAV9-EF1a-Dio-RV-G were all packaged into the 2/9 serotype and tittered at about 3 × 10^12^ genome copies per milliliter. To retrograde trace, the whole-brain mono-synaptic inputs in the OB, a mixture of AAV9-EF1a-Dio-GFP-TVA and AAV9-EF1a-Dio-RV-G (volume ratio: 1:1, 200 nl in total) was injected into the OB of rats, whose coordinates were the same as the *overexpression of* α-Syn experiment. Then, 250 nl of RV-EnvA-ΔG-dsRed was injected 2 weeks later into the OB at the same injection site as the AAV mixture. One week after the RV injection, the animals were perfused for confocal imaging. All viral tools were packaged by BrainVTA (BrainVTA Co., Ltd., Wuhan, China) and all aliquots were stored at − 80 °C.

#### Catecholamine quantification by high-performance liquid chromatography (HPLC)

To detect the level of catecholamine in the striatum-SN system, the independent animals’ model was established as the previous description [32]. Rats(6 rats every group) were sacrificed by deep anesthesia using the pentobarbital sodium (50 mg/kg) and then dissected 12 weeks after AAV injection for overexpression in rats. The striatum samples were frozen in liquid nitrogen to prepare to quantify the catecholamine in the striatum by HPLC analysis. Brain sections were homogenized in 500 μl of 0.1 M TCA (10–2 M sodium acetate, 10–4 M EDTA, 10.5% methanol) as per previously described [32]. Samples were centrifuged at 10,000 g for 30 min to remove the supernatant. Catecholamine levels were analyzed by HPLC coupled with electrochemical detection with an Antec Decade II (Zoeterwoude, Netherlands). Supernatant samples were injected with a water autosampler onto a Phenomenex Nucleosil (5u, 100A) C18 HPLC column (150 × 4.60 mm). Then, samples were eluted with a mobile phase followed by delivery of the solvent at 0.38 ml/min with a Waters 515 HPLC pump. The mobile phase composition was: 75.2 mM sodium phosphate (monobasic, monohydrate), 1.39 mM 1-octanesulfonic acid (sodium salt, anhydrous), 0.125 mM ethylene diamine tetra-acetic acid, 0.0025% triethylamine, and 10% acetonitrile; pH 3.0 adjusted with 85% phosphoric acid. The levels of 3,4-dihydroxyphenylacetic acid (DOPAC), and dopamine (DA) were detected. Waters Empower software was used for HPLC control and data acquisition. Catecholamine values were expressed as ng/mg total protein.

### Behavioral tests

#### Odor discrimination test (habituation/discrimination test)

This test was used to assess olfactory function by habituation/dishabituation in a non-associative memory task. All the odor tests were performed in the home cage to avoid to odor contamination. To investigate the olfactory behavior, a threshold value was tested first. An increasing incremental concentration of lemon (10^− 12^, 10^− 10^ and 10^− 8^) in mineral oil was used to test the odor response by observing sniffing behaviors [33]. A different liquid (50 μl) was dropped onto a swab. When the animal was close to the swab with its nose, the behavior was called a sniff behavior. Then, cross-habituation methods were used to measure non-associative memory [34, 35]. In this test, a rose odor was used as a familiar odor, and a lemon odor was used as the novel odor in this trial [34]. The different odors were dropped onto a swab as the odor emitter, and the number of sniffs each animal made was recorded and counted by an observer blind to the test. First, animals were exposed to the rose odor in consecutive trails (3 min × five times) for the habituating process and then they were exposed once to the novel odor (lemon) for dishabituation (3 min). The olfactory sensory ability of rats was measured by the number of times the rats sniffed the swab.

#### Open field test

The open field apparatus consisted of a square arena (45 × 45 × 40 cm) made of grey polyvinyl chloride plastic boards with a white cross pattern floor and record system (Any maze, Co., USA). The arena was lit by a light-emitting diode light placed 220 cm above the arena. The light intensity was 30 W at the center of the arena. The trials were recorded by a video camera placed 100 cm above the arena. Before the trial, all animals were permitted to habituate to the apparatus for 30 min. For each session, a rat was placed in a particular corner of the arena and allowed to explore for 5 min. During the test session, the total distance traveled and the number of times the white line was crossed in the center of the area were measured automatically using the ANY-maze Video Tracking System. The apparatus was cleaned with 70% ethanol as soon as the test of each animal was finished.

#### Rotarod test

To test the muscular coordination of rats expressing the human alpha-synuclein double mutant, the rotarod test was carried out. It included the cylindrical arrangement of thin steel rods, 75 mm in diameter, which was divided into two parts by compartmentalization to permit the testing of two rats at a same time. Before the start of the test, rats were trained on the rotarod apparatus until they stayed on the rod for at least the cut-off time. During the training, the speed was set at ten cycles per min and cut-off time was set at 3 min. First, the rats were allowed to remain stationary for a while and then the rotational speed was steadily increased by 10 rpm in 20 s intervals until the rats fell off the rungs. Animals were tested for two trials per day, and the mean duration time the rat stayed on the rod was recorded [36].

#### Preparation of the brain tissue and pathological evaluation

All the rats were anesthetized with 400 mg/kg chloral hydrate (4% in saline, 5 ml/kg) and perfused them transcardially with 0.9% saline, followed by 4% PFA in phosphate buffer (pH = 7.2) for histological experiments. After perfusion, brain tissue was placed in 4% PFA for 4 h and then was dehydrated by gradient sucrose in phosphate buffer (10%, 20%, and 30%) until the brains completely sank to the bottom. The entire brain of each rat was cut into the coronal sections (25 μm) on a freezing microtome, and stored at − 20 °C.

#### Immunohistochemistry and immuno-fluorescence

GFP labeling was performed to detect viral over-expression and to trace transferring and aggregation of hm-α-syn from the OB to other brain regions. Immunohistochemistry was used to detect the endogenous α-syn (Abcam, ID: ab27766) and tyrosine hydroxylase (TH). A standard peroxidase-based method (Vectastain ABC kit and DAB kit; Sigma, ID: A2054) was used in these processes. To stain coronal free-floating sections, primary antibodies anti-rat α-syn (monoclonal raised in mouse, 1:500, Abcam) or anti-TH (raised in rabbit, 1:1,000, Abcam), anti-alpha-synuclein (phospho S129) (ab51253, monoclonal raised in rabbit, 1:1000), Anti-LC3B (raised in rabbit, 1:500, stock number: ab63817) and biotinylated secondary antibodies (sheep anti-mouse, 1/200, Vector Lab; Donkey anti-rabbit 1/200, Abcam) were used. These sections were analysed by conventional microscopy (BX43, Japan) and confocal microscopy (FV10i, Olympus, Japan). Images were captured with a VS120 digital camera using VS120ements AR 4.00.08 software (Olympus). The presence of positive cells was assessed in a blinded manner by screening every single section at 20× magnification.

### Golgi staining

The rapid Golgi staining kit (GolgiStain™ Kit, Neurotechnologies, Inc.) was used to stain the pyramidal neurons in the different brain fields. In these studies, the Golgi staining was selected to investigate the qualitative and morphometric properties of neurons in various areas. Before brain tissue treatment, slice sections were treated twice to create coated gelatin-dipped slides and allowed to air-dry at room temperature in the dark. Brain tissues were treated as previously described [37, 38]. In brief, after anesthesia (0.3 mL 4% chloral hydrate per animal, Henry Schein, Inc.), brains were immediately removed, rinsed with deionized water, and dropped into a Golgi box solution containing mercuric chloride, potassium dichromate, and potassium chromate. The brains were stored at room temperature for 21 days in the dark. Then, the brains were transferred to a cryoprotection solution for 1 week in the dark and sectioned coronally at a thickness of 200 μm with a cryostat. The sections were rinsed in distilled water (3 min × 3). Then the sections were dehydrated in 50, 75, 95, and 100% ethanol; cleared in the TO bio-clarifier (5 min × 3) and cover-slipped with the resinous mounting medium. ImageJ for the Windows system (NIH: 1.6.0_24) was used to analyze the difference in the dendritic and spine morphology between groups by two observers blinded to the experimental conditions. For analysis of dendritic spines, entirely visible spines with minimal obstruction from neighboring Golgi-stained cells were used for quantitative analysis (100 × oil immersion lenses). For each brain field, 15 neural cells were selected to be evaluated by Sholl analysis, dendritic arbors of at least 30 pyramidal neurons from each animal were traced at high magnification. Dendritic-spine number, length, and dendrite diameter were counted over 20 μm lengths at the beginning of the dendrites of pyramidal neurons. Spine density was expressed as the average number of spines per micron of dendritic length.

### Transmission electron microscopy (TEM)

An electron microscope was used to observe the ultrastructure of autophagosomes. Animals were sacrificed 12 weeks after being administered the AAV injections in the OB (*n* = 4). Fixed brain tissues samples from each group were sliced with a microslicer and were fixed in 3% solution of glutaraldehyde (stock No. G5882; Sigma-Aldrich, USA) in 0.1 M cacodylate buffer (pH = 7.4, stock No. G20840; Sigma-Aldrich, USA) at 4 °C overnight. After osmification, the samples were dehydrated by the gradient ethanol, cleared in propylene oxide (stock No. G56671; Sigma-Aldrich, USA) and then embedded in Epon (stock No. G45347; Sigma-Aldrich, USA). After dehydration, sections were stained with Toluidine blue and analyzed by an Olympus BX41 light microscope (Olympus, Japan).

### Double staining

#### Thioflavin-S(ThS)/ p-α-Syn 129 staining

Free-floating brain tissue slices were washed with 0.1 M PBS (3 min × 3), then mounted onto slides, air-dried and then rehydrated with ultrapure water. Sections were stained with 0.1% Thioflavin-S ethanol/PBS for 10 min. After washing with 0.1 M PBS (3 min × 3), the sections were incubated with primary antibody anti-α-synuclein (phospho S129) (ab51253, monoclonal raised in rabbit, 1:1000) overnight, and then with Donkey anti-Rabbit IgG(ThermoFisher, Alexa Fluor 594, Catalog # A-21207). Slides were then mounted using Vectashield (Vector Laboratories).

#### LC3b/TUNEL staining

To explore if neurons undergoing autophagy degenerate in association with apoptosis, LC3b and TUNEL *(terminal deoxynucleotidyl transferase-mediated dUTP nick end labeling)* staining was performed to illuminate this relationship. TUNEL staining was performed as previous described [39]. Free-floating brain tissue slices needed to be rehydrated in the cryostat for 10 min in PBS followed by washing with DNase-free water for 5 min at room temperature. Then sections were incubated in Proteinase K solution for 30 min at room temperature. After washing (3 min × 3) in DNase-free water, the endogenous peroxidase activity of these slices was blocked by H_2_O_2_ for 10 min. Next, the slices were incubated in TdT labeling buffer for 5 min and then TdT labeling mixture for 2 h at 37 °C with blocking reagent at room temperature for *30 min.* After TUNEL staining, slices were washed with 0.1 M PBS (3 min × 3), the samples were blocked with donkey serum for 30 min and then incubated with primary antibodies (anti-LC3B, raised in rabbit, 1:500, stock number: ab63817) overnight. After washing (3 min × 3), the slices were incubated with the second antibody (conjugated to Alexa Fluor 488, Abcam, #ab150073) and mounted using Vectashield.

### Statistical analysis

Before all data were analyzed, the obtained data were evaluated to determine if there was a normal distribution. Behavioral data were analyzed by an unpaired Student’s *t*-test or repeated-measure analysis of variance (ANOVA) and represented as the mean ± standard error (mean ± SEM) in SPSS 13.0 software (USA). Immunohistochemical data were analyzed by an unpaired Student’s *t*-test and represented as the mean ± standard deviation (mean ± SD). The threshold value for acceptance of differences was 0.05. Origin 8.0 was used to present the results.

## Results

### Identification of AAV hm-α-Syn expression in the OB

To investigate the expression of AAV-hm-α-syn in the OB, sections of the OB were examined to confirm the location of the AAV injection. Animals with inaccurate injection locations were excluded. Also, the expression of GFP was used to confirm the expression of hm-α-syn or control GFP (AAV-GFP) in the OB. GFP-immunoreactive signals were detected in both the mitral cell bodies and neurites of the OB of rats injected with AAV-hm-α-syn and with the control AAV (Fig. 1b). No difference in GFP labeled cell numbers between these two groups was observed 3 weeks after the injection (Fig. 1c). However, hm-α-syn expression resulted in stronger GFP labeling in the cellular processes.

**Fig. 1:** Identification of AAV hm-α-Syn expression in the OB. **a** Nissl stained section showing an example of the OB injection. Arrows point to the precise location of the site of the needle tract. **b** Representative examples of the GFP labeling patterns from the AAV-hm-α-Syn-GFP and control AAV-GFP injection animals. **c** Comparison of the numbers of GFP positive cells between the AAV-hm-α-Syn-GFP and control AAV-GFP injected animals

### Detection of hm-α-Syn in brain regions beyond the OB

The areas of GFP-positive signals were mapped in the whole brain to determine the extent of hm-α-Syn-GFP spread after the AAV injection (Fig. 2). In the AAV-hm-α-Syn-GFP group, GFP labeling was found in the OB, the AON (anterior olfactory nucleus), the prepiriform cortex (PPiri), the CPU (caudate-putamen of the striatum), and the SN (substantia nigra). In the control group, the GFP labeling was only found in the OB, the AON, and the PPiri. No GFP^+^ cells were found in the nigrostriatal system. These results indicate that both the hm-α-Syn-GFP and the control GFP were expressed in the olfactory fields by the AAV, but only the hm-α-Syn-GFP was transferred to the adjacent brain regions.

**Fig. 2:** Hm-α-syn was detected in brain regions beyond the OB 3 weeks after the AAV injection. Representative examples of high magnification images (scale bar: 20 μm) of the OB, the AON, the PPiri, the CPU, and the SN are shown. No GFP signal was found in the SN in the control animals. Arrows point to GFP positive cells (bar: 20um)

### Monosynaptic projections from the striatum and SN cannot reach the OB field

A retrograde viral vector, pseudorabies viral GFP (RV), was used to trace projections from outside structures that reached the OB and to determine the structural basis upon which hm-α-syn was transferred between cells. The signals of the RV tracing was examined in the OB, the AON, the Piri, and the CPU. The experiments found that there were signals in these sections (Fig. 3), indicating that mitral cells in the OB receive projections from these brain regions, as supported by previous studies [34, 40].

**Fig. 3:** Representative retrograde labeling in brain regions following RV infection in the OB. Signals from RV were detected in α-syn-positive fields including the OB, the AON, the Piri, and the CPU 3 weeks after the AAV injection. No projections from the SN were found

### AAV-hm-α-Syn induces a loss of dopaminergic neurons and DA levels in the striatum-SN system

The number of TH^+^ cell bodies and fibers in SN-striatum field in hm-α-syn rats vs. control rats 12 weeks after AAV injection was contrasted to study if hm-α-syn overexpression contributed to the destruction of dopaminergic neurons in the SN. Results (Fig 4b and c) show that there was a definite decrease in TH^+^ neuronal cells bodies of the SN (SN: 12 w, *p* < 0.05) and in fibers of the striatum (striatum: 12 w, *p* < 0.01) after AAV injection. Together with a previous report [41], these data suggest that the hm-α-syn overexpression induced the loss of the cell bodies and nerve terminals in dopaminergic neurons of the substantia nigra.

**Fig. 4:** Effect of AAV-hm-α-syn injection on the number of dopaminergic neurons *and DA levels* in the striatum-SN. **a** Presentation of the TH-positive cells in the striatum and SN 12 weeks after injection into the OB. **b** & **c**) Comparison of the TH-positive cells in the SN and fibers in the striatum 12 weeks after injection into the OB. These results indicate that the number of TH-positive cells bodies and terminals in the SN-striatum fields is reduced 12 weeks after AAV-hm-α-syn injection. *P < 0.05, **P < 0.01. **d** & **e**) Comparison of DA and DOPAC level in the striatum. These results indicate that DA and DOPAC level in the SN-striatum fields is reduced 12 weeks after AAV-hm-α-syn injection. *P < 0.05, **P < 0.01. All data are presented as mean ± SD. (Bar: 20um)

At the same time, the HPLC (Fig 4d and e) was performed and analyzed for DA and the metabolite DOPAC to further evaluate dopaminergic neurotransmitter and metabolite levels in the striatum system. A significant reduction of striatal DA levels is to 50% relative to the control group (*p* < 0.01) and striatal DOPAC levels to 44% compared to the control group (*P* < 0.01) was found 12 weeks after the AAV injection in the OB. Thus, the AAV-mutant-alpha-synuclein overexpression was found to significantly decrease DA and DOPAC levels of striatum in comparison to the control injection.

### Mutant α-syn injected in the OB induced increases of pSer129 α-syn in multiple brain regions

Posttranslational modification of α-syn was thought to influence its aggregation and found in more than 90% of LB formations [12, 42]. Phospho-Ser129 α-syn^+^ cells were examined 12 weeks after AAV injection to determine whether the mutant α-syn in the OB induced α-syn aggregation in the brain (Fig. 5a and b). The experiment found that the number of pSer129 α-syn positive cells was significantly increased in AAV-hm-α-syn injected animals in comparison to the controls (*p* < 0.05) in the OB, the AON, the PPiri, the PFC, the LS, the Cpu, the Hip, the LG, the VTA, and the SN (Fig. 5a). These results demonstrate that human mutant α-syn in the OB induced α-syn aggregation in adjacent brain regions, which extended beyond the regions of hm-α-syn expression.

**Fig. 5:** AAV-hm-α-syn injected in the OB increased pSer129 α-syn in multiple brain regions. **a** Expression of hm-α-syn in the OB increased the level of pSer129 α-syn in multiple-brain regions. OB, olfactory bulb; AON, anterior olfactory nucleus; Piri: piriform cortex; PFC: prefrontal cortex; LS: lateral septal nucleus; CPU: caudate putamen; Hip: hippocampus; LG: lateral geniculate nucleus; VTA: ventral tegmental area; SN: substantia nigra. **b** Comparing a number of the pSer129 α-syn^+^ cells between the experimental and control animals. Error bars represent mean ± SD, *n* = 8. Statistical comparisons were performed using the student’s test, *p < 0.05. (Bar: 20um)

### Progressive olfactory deficits and motor impairment after AAV-hm-α-Syn injection

Incremental increasing concentrations of rose (10–12, 10–10 and 10–8) in mineral oil (solvent) were used to study olfactory-related behaviors in the rats. The experiments found that AAV-hm-α-syn injection in the OB induced olfactory responses at 10^− 8^ concentration of lemon (Fig. 6a), whereas control animals responded to 10^− 10^ and 10^− 8^ concentrations. In subsequent examinations, the 10^− 8^ concentration was used to conduct an olfactory discrimination test 3, 6, 9, and 12 weeks after the animals were injected with the AVV-hm-α-syn vector; they animals were habituated with five trials of rose smelling sessions to reduce their sniffing of this odor. They were then exposed to 10^− 8^ concentration of lemon odor. While control animals were able to identify by sniffing this new odor, the hm-α-syn mice sniffed significantly less at the new odor (Fig. 6b).

**Fig. 6:** Rats injected with the AAV-hm-α-syn exhibit progressive impairment in odor discrimination and motor behaviors. **a** Animals were exposed to the 10^− 8^ rose odor for consecutive trials (habituation) and then exposed to increasing concentrations of lemon in mineral oil (10^− 12^, 10^–10,^ or 10^− 8^ unit) for three consecutive trials (dishabituation) to test the response threshold after the AAV injection. # means a significant difference (*p* < 0.05) contrasted with the last test in the habituation (oil 3). **b** Results of the odor habituation/dishabituation test. After the habituation trials for sniffing rose odor, rats showed impaired odor habituation/dishabituation behavior 3 weeks after AAV-hm-α-syn injection than control. Also, 6, 9 and 12 weeks after the AAV-hm-α-syn injection (**c** and **d**) in the OB, locomotion in the open field was reduced. The number of times crossing the line and the total distance traveled were lower 6 weeks after the AAV-hm-α-syn injection. The rod test showed that 12 weeks after AAV hm-α-Syn injection in the OB, the rats had decreased the amount of time they stayed on the rod relative to control treatment. Data are presented as mean ± SEM. *P < 0.05, **P < 0.01. **e**. Latency time 12 weeks after AAV injection of OB (*n* = 8/group). The values are presented as mean ± standard deviation (SD)

AAV-hm-α-syn injection in the OB also impaired motor activity in the open field test. The number of times line crossing was decreased 6 weeks after the AAV-hm-α-syn injection (Fig. 6c and d; hm-α-Syn vs. control, 3 weeks: *p* > 0.05; 6 weeks: *p* < 0.05; 9 weeks, *p* < 0.05 and 12 weeks *p* < 0.05). Significant decreases were found in the total distance traveled in the open field of the rats treated with AAV-hm-α-syn (hm-α-Syn vs. control, 3 weeks: *p* < 0.05; 6 w: *p* < 0.05; 9 w, *p* < 0.05 and 12 w *p* < 0.05).

For muscular coordination ability, a rotarod test was used to measure the muscular coordination in the PD rat model [43]. As shown in Fig. 6e, 12 weeks after AAV-hm-α-syn injection, the animals displayed the decreased times staying on the rod compared with the control group (*p* < 0.05). Taken together, these results show that injecting AAV-hm-α-syn into the OB induced dysfunction in the olfactory discrimination task, in locomotor activity, and in muscular coordination in comparison to the control rats.

### Density and morphological distribution of dendritic spines in sensitive brain fields identified by Golgi staining

Twelve weeks after the AAV injection into the OB, the density and morphological distribution of dendritic spines in multiple brain regions, including the OB, prefrontal cortex (PFC), hippocampus (Hip) and striatum caudate putamen (CPu) were investigated by Golgi staining to explore pathological changes in spine and dendritic protrusions (Fig. 7). Significant morphological changes were found. Reduced spine density was seen in the SN (Fig. 7a). It was found (Fig. 7c and d) that there were fewer branches in several brain regions in the rats injected with AAV-hm-α-syn than in the controls (OB: *p* < 0.05; PFC, *p* > 0.05; Hip, *p* < 0.05; and CPU, *p* < 0.05). Sholl analyses of the density of dendritic spine in these brain regions displayed impaired protrusion density. There was a significant decline in dendritic protrusions compared to controls 12 weeks after AAV injection (vs. control, OB: *p* < 0.05; PFC, *p* < 0.05; Hip, *p* < 0.05; CPU, *p* < 0.05). These findings were consistent with previously published findings on α-syn effects [41].

**Fig. 7:** Golgi staining identified the effect of AAV-hm-α-syn injections on neuronal morphology. (**a** and **b**) Representative photographs of dendritic protrusions in the substantia nigra. A: 20× magnification. B: 100× magnification in oil immersion. (**c**) Effect of AAV-hm α-syn on spine density. These results indicated that there was a more significant decrease in spine density in several brain regions in rats injected with AAV-hm-α-syn (vs. control, * means *p* < 0.05). **e** Representative photographs of dendritic spines in the SN (100× magnification times in oil immersion). **d** Effect of AAV-hm-α-syn on the total number of intersection points. The results indicated that there was a significant reduction of the total number of intersection points in different brain regions in rats treated by AAV-hm-α-syn (vs. control, * < 0.05). Data are presented as mean ± SD. *P < 0.05, **P < 0.01. **f**: Representation diagrams about Goligi staining by AAV & control injection

### AAV-hm-alpha-Syn induced autophagy in sensitive fields of rat brain tissue

Autophagy has been associated with symptoms in PD. Interestingly, intracellular α-syn protein has been reported to be related to neuroprotection against autophagy, whereas mutant α-syn inhibits intracellular degradation of misfolded proteins [44]. An autophagic marker, LC3B, was measured in the OB and SN (Fig. 8) to further explore the reasons behind the decrease in a number of dopaminergic neurons. After the AAV- hm-α-syn injection, the relative number of the LC3B-positive cells increased significantly. The mutant α-syn caused a significantly more LC3B increase than controls (*p < 0.05).

**Fig. 8:** The effect of AAV-hm-α-syn injection on the number of LC3B-positive cells in the OB and SN. (**a**) Representative microphotographs of TH-positive cells in OB and SN from rats 6, 9 and 12 weeks after AAV-hm-α-syn injection into the OB. LC3B-positive cells in the OB and SN from 6, 9 and 12 weeks after the injection into the OB. (**b**) These results indicated that the number of LC3B-positive cells in the OB and SN field was enhanced 6weeks to 12 weeks after the AAV-hm-α-syn injection. Data are presented as mean ± SD. *P < 0.05, **P < 0.01. (Bar: 20um)

### The number of autophagic vacuoles increased in the OB and SN of rats 12 weeks after the AAV-hm-α-syn injection

The formation of autophagosomes in the OB and SN neurons was explored using electron microscopy (EM). Autophagosomes were visible in the OB and SN neurons of rats 12 weeks after the AAV-hm-α-syn injection (Fig. 9). EM revealed that there were more autophagosomes in the OB and SN 12 weeks after the AAV-hm-α-syn injection in comparison to control rats. The size of the autophagosomes was also larger.

**Fig. 9:** A comparison of the ultrastructural examination of autophagosomes in the OB and SN of AAV-hm-α-syn and control animals. 12 weeks after the AAV injections, representative electron micrographs were acquired from rats. Scale bars: 500 nm

### Immunofluorescence double staining

Immunofluorescent double-labeled staining was used to further explore the neuronal mechanism of hm-α-synuclein pathology in the rats. First, LC3B and TUNEL staining were performed to determine if autophagy neuron degeneration was associated with apoptosis. The cortex of substantia nigra (SN) was selected to evaluate this association. It was found that many cells were labeled by LC3B (green) and that some of the LC3B positive cells were co-localized with TUNEL staining (red) in the hm-α-synuclein rats (Fig. 10). The TUNEL stain is a method for detecting DNA fragmentation by labeling the 3′- hydroxyl termini of double-stranded DNA breaks generated during apoptosis. However, lower co-localization was found in the controls. This indicates that the apoptosis happened in some cells overexpressing the hm-α-synuclein. Second, double-labeling was used to determine if phosphorylated-Ser129-alpha-synuclein (pSer129 α-synuclein) was co-localized with markers of Lewy body formation. Thioflavin-S, a positive marker of Lewy bodies (green), and pSer129-α-synuclein (red) were used to detect further pathology. More double-labeled cells (yellow) were found in the hm-α-synuclein injected rats than in control treatments. This data indicated that the pSer129-α-synuclein signals reflected LB pathological changes.

**Fig. 10:** Immunofluorescent double-labeled staining in the SN field. **a**-**c** double staining of SN field by LC3B (green) and TUNEL staining (red) in the control rats. **d**-**f** double staining of SN field by LC3B (green) and TUNEL staining (red) in the hm-α-synuclein rats. These data indicates that the apoptosis happen in some cells overexpressing the hm-α-synuclein. **g**-**i** double staining of SN field by ThS (green) and pSer129-α-synuclein staining (red) in the control rats. **j**-**l** double staining of SN field by ThS (green) and pSer129-α-synuclein staining (red) in the hm-α-synuclein rats. These data indicates that pSer129-α-synuclein signals reflected LB pathological changes. (Bar: 20um)

## Discussion

Parkinson’s disease is a common degenerative disease. However, there remains a need for accurate animal models to investigate mechanisms that underlie the prodromal phase of the disease. This lack of accurate modeling systems limits the development of early diagnostic tools and effective treatments. This study aimed to generate a rat model for PD that develops behavioral deficits and histopathological hallmarks resembling the human disease. Previous studies have reported that α-syn plays a vital role in PD initiation and that olfactory dysfunction is often found in the early phase of PD [17, 21, 45]. In the current study, the local overexpression of hm-α-syn in the OB was used to trigger α-synucleinopathy in the rat. Three weeks after hm-α-syn vector administration, the hm-α-syn, which was fused to GFP, was found over a wider range within the brain. The hm-α-syn was found gradually from the OB to multiple olfactory and non-olfactory brain regions. Mutant hm-α-syn was found in the substantia nigra field, which is a recognized area damaged in the PD development process [46]. After 12 weeks, pSer129-α-syn-positive cells and hm-α-syn positive cells were found in many brain regions. These cells overlapped in some areas, but the pSer129 α-syn-positive cells were observed in more widely distributed brain regions than hm-α-syn positive cells.

Further studies suggested that pSer129 α-syn was found in LBs, which is a marker of PD, and that hm-α-synuclein expression also enhanced autophagy. The double staining found that the LC3B that was a marker of autophagy colocalized with the apoptosis marker that was mapped by the TUNEL staining. These findings partly explain the increased apoptosis in the hm-α- positive synuclein cells. The results also revealed that there were pathological changes beyond the spread of the hm-α-syn positive cells. In the morphological evaluation, dendritic protrusion density and morphology were subsequently analyzed in different brain regions. This evaluation found that both dendritic protrusion density and neural branch number were decreased in the AAV-hm-α-syn injected animals in comparison with controls.

Furthermore, the results revealed that the number of dopaminergic neuronal body and fibers in the SN was decreased. In the behavioral tests, olfactory discrimination ability was found that to be impaired 3 weeks after the AAV-hm α-syn injection. In the open field test, the total distance traveled by the AAV-hm α-syn injected animals was reduced after 3 weeks and the number of times crossing the line was reduced after 6 weeks. In general, these results not only mimicked the transfer of α-syn between cells but also demonstrated that hm-α -syn induced phosphorylation of normal endogenous α-syn, potentially propagating α-syn aggregation (namely LB formation) and leading to neuronal damages in the SN.

### Human mutant α-syn in the OB was found with a wider scope along anatomical pathways and induced Lewy body pathology

Clinical studies have suggested that PD symptoms, including motor and non-motor symptoms, need to be considered as a severe multi-system neurodegenerative disorder [47, 48]. The motor symptoms of Parkinson’s disease (PD) including bradykinesia, muscular rigidity, and tremor depend upon the degeneration of the dopaminergic neurons in the substantia nigra pars compacta [49]. As such, motor symptoms originally derive from the selective damage of dopaminergic neurons in the mesencephalon. Non-motor symptoms of PD are originally from neuropathological alterations outside the substantia nigra and are found earlier than motor-symptoms in the clinic. As such, non-motor symptoms are recognized as prodromal symptoms of PD [50]. Autonomic disturbances, olfactory dysfunctions, depression and sleep disorders may represent prodromal non-motor symptoms of PD [51, 52]. In our study, olfactory impairment was found 3 weeks after AAV-hm-α-syn injection; motor ability impairment was found 6 weeks after and decreased muscular coordination (i.e., balance on the rotarod) was found 12 weeks after. Recent neuropathological studies indicate that Lewy bodies accumulation in several neuronal cell types in the brain can be used as an intraneuronal landmark of PD because LB formation has been reported widely, from the medulla oblongata and olfactory bulb to neocortical areas [53]. As such, the PD model developed here is by previously reported animal models [2, 48, 54] because the mutant α-syn overexpression in the olfactory bulb mimicked prodromal symptoms of PD. Further evaluation of this model may contribute to the development of the precocious diagnosis of PD and may be used in the future to test the efficacy of neuroprotective agents.

Human mutant α-syn protein was expressed in the OB by an AAV expression vector. This mutant protein was fused with GFP as a marker to trace the position of hm-α-syn. Previous studies on cell-to-cell transmission of misfolded preformed fibrils (PFF) of α-synuclein (α-syn) often used pSer129 α-syn-positive detection as a method to trace exogenous synuclein [10, 41]. Abnormal aggregation of α-syn within neuronal perikarya (Lewy bodies) and neurites (Lewy neurites) are defined as neuropathological hallmarks of Parkinson’s disease [53]. The inclusions found in this study have a tendril-like cytoplasmic structure around the nucleus that was similar to previous studies induced by fibril synuclein [41].

Moreover, this study showed that human mutant α- synuclein overexpression in the OB induced pSer129 α-syn expression in a much wider scope beyond the injection site. This scope of pSer129 α-syn is often viewed as a pathological marker and is implicated in the pathogenesis of Parkinson’s disease [55, 56]. For example, there is a correlation between pSer129-α-synuclein concentrations in the cerebrospinal fluid (CSF) of PD patients and UNIFIED PARKINSON’S DISEASE RATING SCALE (UPDRS) scores [57].

Regarding the pathogenic mechanism hm-α-syn injection, previous studies found that injected hm-α-syn co-localized with pSer129 α-syn-signals [58, 59]. Our study confirmed that pSer129 α-syn-signals are found in LBs, which is an important biomarker of PD, and that the scope of pSer129 α-synuclein signals was wider than LBs in the model. Therefore, it was speculated that pSer129 α-synuclein might be a vital molecule that ultimately aggregates into LB. It is important to note the human α-syn used in this experiment was fused with GFP, which may affect the α-syn structure. This change makes the transfer of injected hm-α-synuclein different from that of native α-syn.

Moreover, the distribution of pSer129 positive cells is wider than that of GFP-positive cells. At the same time, experiments investigating monosynaptic connections to the OB using an RV tracer showed that brain regions labeled in the controls included the AON, Piri, and CPU, but not the SN, which was consistent with an earlier study [60]. Taken together, it is concluded that the hm-α-syn injected into the OB transferred beyond the monosynaptic connections because the presence of hm-α-syn and pSer129 hm-α-syn had a broader distribution pattern than the viral vector alone, which is indicative of a downstream pathology related to the expression of the mutant hm-α-syn protein within the olfactory system.

### (aSyn PFF)

Previous studies have reported that α-syn forms the pre-formed fibril α-syn(PFF) of relatively uniform size when treated by sonication and that this α-syn PFF seed the recruitment of endogenous α-syn within 3–5 days to form aggregates characterized by detergent-insolubility and hyperphosphorylation in vitro [61]. However, in vivo studies have shown that fibril α-syn does not induce pathological changes until 3 months after injections in the OB [41]. In contrast, the experimental model presented here based on hm-α-syn injection in the OB produced pathological changes over a much shorter time frame.

An analysis of olfactory and motor functions was included in this study to assess behavioral effects in the model. The experiments showed a progressive and specific deterioration of olfactory function, which was similar to olfactory deficits seen in early clinical stages of PD before motor dysfunction [62, 63]. Odor discrimination ability was slightly impaired 3 weeks after hm-α-syn injection, but severe dysfunction developed within 12 weeks after the injection. In the motor function analysis, clear evidence of physiological damage was reflected in the total distance traveled and a number of times crossing the line after hm-a-syn administration. In the control test, no dysfunction was found in the behavioral evaluations, which indicates the olfactory and motor functions deficits observed were the result of the mutant hm-α-syn administered to the OB.

### Dopaminergic cells loss and dopamine neurotransmitter decrease in the SN-striatum field

Parkinson’s disease is a neurodegenerative disorder characterized by the progressive loss of dopaminergic neurons in the substantia nigra [3]. It was found in this study that the number of TH-positive cell bodies and fibers was significantly decreased in the striatum and SN fields. With regards to the dopamine neurotransmitter, both decreased levels of DA and DOPAC were found in the animal model, which is accordant with previous studies [2]. Further data indicated that there were autophagic responses in sensitive brain regions as an increased number of LC3B positive cells were identified. Some of these LC3B positive cells were co-localized with TUNEL assay signals indicating that apoptosis took part in the dopaminergic cell loss process [64]. Autophagy and apoptosis are basic physiological processes that contribute to cellular homeostasis. Autophagy is a process clearing long-lived cytosolic proteins and damaged organelles from the cell. Apoptosis is a form of programmed cell death controlling cellular homeostasis [65]. It is thought that as hm-α-syn begins to express in some cells, a stress response is induced leading to autophagy response enhancement. When mutant α-syn aggregates in cells, the toxic effects of aggregation inhibit autophagy leading to apoptosis [65, 66]. The results of Thioflavin-S staining indicated that there were much more Th-S-positive cells in sensitive brain areas following hm-α-syn injection. This suggests that different autophagy processes were found in the experiments and that further experiments are needed to explore the long-term effects of the hm-α-syn on autophagy and apoptosis.

### Hm-α-syn induced pathological changes at the morphological level

In the morphological analysis evaluated with Golgi staining, immunohistochemistry and ultrastructural examination, the density and morphological distribution of dendritic spine in several brain regions, including the OB, prefrontal cortex (PFC), hippocampus (Hip) and striatum caudate putamen (CPU), were found to be altered 12 weeks after hm-α-syn injection in the OB (Fig.5). There were fewer branches in these brain regions after hm-α-syn injection. The density of dendritic spines in these brain regions exhibited lower protrusion density, and there was a significant decline in the number of dendritic protrusions 12 weeks after AAV injection. Previous researchers have demonstrated that the density of dendritic spines and morphological distribution reflects pathological changes in PD [67, 68]. Golgi staining has been compared with neural staining and was found to slightly underestimate the density of dendritic protrusions in the neuron [69]. Moreover, some protrusion morphology was not detected in our experiments due to the resolution of the light microscope (0.2 μm in the horizontal plane and 0.8 μm in the vertical plane) because the better resolution of light microscopy is needed for their detection. Maintenance of axon and dendrite length is critical for neuron function, and autophagy is actively involved in regulation of pathological remodeling.

## Conclusion

The results presented here suggest that the overexpression of mutant α-syn obtained with AAV–hm-α-syn vector can transfer among cells and induce Lewy body formation in relevant brain regions, leading to impairment of behavioral functions related to both motor and non-motor systems. In general, the olfactory bulb is a special site that is susceptible to pathogenic factors including mutant α-syn. However, further work is needed to understand the involvement of olfactory regions in PD development. Together, this experiment demonstrated a novel and valid model of prodromal PD.
